This article has been retracted.

# Research on Early Warning Mechanism and Model of Liver Cancer Rehabilitation Based on CS-SVM

**DOI:** 10.1155/2021/6658776

**Published:** 2021-01-12

**Authors:** Bo Jianzhu, Li Shuang, Ma Pengfei, Zhu Yi, Zhang Yanshu

**Affiliations:** ^1^School of Public Health, North China University of Science and Technology, Tangshan, 063021, China; ^2^Laboratory Animal Center, North China University of Science and Technology, Tangshan, 063021, China; ^3^School of Science, North China University of Science and Technology, Tangshan, 063021, China

## Abstract

Since the 20^th^ century, cancer has become one of the main diseases threatening human health. Liver cancer is a malignant tumor with extremely high clinical morbidity and fatality rate and easy recurrence after surgery. Research on the postoperative recurrence time and recurrence location of patients with liver cancer has a crucial influence on the postoperative intervention of patients. Evaluation of the clinical manifestations of patients after liver cancer surgery is conducted according to medical knowledge or national standards to determine the main factors affecting liver cancer rehabilitation. In order to better study the mechanism of liver cancer recurrence, this paper uses CS-SVM to predict the recurrence time of liver cancer patients, so as to timely intervene the patients. There are five evaluation indicators which are basic indicators, immune indicators, microenvironment indicators, psychological indicators, and nutritional indicators, respectively. This paper collects the clinical evaluation data of postoperative follow-up visits for patients with liver cancer in a hospital, improves the parameter selection process of the support vector machine by using the search ability of the cuckoo algorithm, and establishes an algorithm-optimized prediction model of support vector machine for the prognosis of liver cancer to predict the location and approximate time of recurrence. According to the clinical evaluation data of patients with liver cancer after surgery, logistics regression, BP neural network, and other related methods are used to predict the prognosis of liver cancer patients after surgery. The prediction effects of several methods are compared, and the superiority of the model is discussed. At the end of this article, we conducted an empirical analysis on the clinical evaluation data of patients with liver cancer after surgery. For the collected samples of 776 liver cancer recurrences after surgery, the established liver cancer prognosis outcome prediction model was used to predict the recurrence time and recurrence location, respectively. The mean square error of recurrence time prediction is 9.2101, which is much smaller than the prediction mean square error of BP neural network of 177.9451; the prediction accuracy of recurrence location is 95.7%, which is much higher than the 63.14% of logistic regression. The empirical analysis results show that the improved support vector machine model based on cuckoo established in this paper can effectively predict the time and location of cancer recurrence.

## 1. Introduction

Cancer has become one of the major diseases that affect human health. It is the main culprit that causes most families to fall into poverty and return to poverty due to illness and seriously affects economic development [1–3]. In recent years, the problem of population aging in developed countries and some developing countries in the world has been growing more and more serious year by year. Coupled with the influence of factors such as environment and lifestyle, the overall incidence and mortality of cancer have been increasing year by year [4].

Liver cancer is a malignant tumor with extremely high incidence and fatality rate. In recent years, the number of liver cancer patients has increased rapidly. Cancer patients are at risk of recurrence after surgery. The evaluation of patients and the mining and analysis of evaluation data through machine learning algorithms will play a pivotal role in the diagnosis, disease progression, and postoperative monitoring of liver cancer patients [5, 6].

In recent years, machine learning (ML) has developed rapidly and has made great achievements in the field of disease diagnosis and treatment and prognosis. Artificial neural networks, support vector machines (SVMs), etc have been widely used in the study of cancer diagnosis, treatment, and prognosis.

When liver cancer recurs after the surgery of a patient, the established liver cancer early warning diagnosis model can be used to predict the future recurrence time and location, which can assist the doctor in diagnosis, and work out a reasonable rehabilitation plan based on various evaluation indicators to improve the survival rate of liver cancer patients. The research results of this article can be extended to the early warning diagnosis of other cancer diseases and improve the recovery rate of cancer patients. It has great significance in the fields of nursing rehabilitation and clinical diagnosis.

Wen et al. [7] calculated the decline rate of CA-199 to predict the postoperative prognosis of breast cancer patients, and related indicators and overall survival time were statistically significant. Li et al. [8] used logistic regression to study the factors affecting the prognosis of patients with liver cancer and found that factors such as patient pathological types were significantly related to the survival time of patients with liver cancer. Wu et al. (2018) [9] studied the effect of serum miRNA-10b on the early recurrence and metastasis of breast cancer after surgery and found that the control group and the recurrence and metastasis group have significant differences and that serum miRNA-10b can be used as a predictive factor for recurrence of breast cancer after surgery. Cheng [10] applied data mining to breast cancer recurrence prediction and analyzed the pros and cons of the C4.5 algorithm, naive Bayes algorithm, and SVM algorithm in breast cancer recurrence prediction. Li et al. [11] proposed a multiclass support vector machine recursive feature elimination method (MSVM-PFE), which was applied to predict the recurrence of liver cancer after surgery and showed high accuracy.

Weiser et al. (2008) [12] used Cox regression to evaluate prognostic factors through multivariate analysis and used cubic splines to model nonlinear continuous variables. The model was bootstrapped internally and verified through consistency index and calibration. The curve evaluates performance and improves the accuracy of colon cancer recurrence prediction. Zhang et al. (2015) [13] discussed the application of multiple biomarkers in the combined detection of liver cancer after rehabilitation, indicating that AFP-L3 plays an important role in the prediction of liver cancer recurrence. AFP-L3 can be used as an indicator to identify benign or malignant liver disease and the risk of recurrence after radiofrequency ablation. Zhou [14] proposed a liver tumor segmentation method based on a three-stage hybrid support vector machine (HSVM). The method can help radiologists identify liver cancer on the basis of multiphase CT images and have a certain positive effect on early diagnosis of patients.

A machine learning algorithm based on structural risk minimization has better generalization ability [15]. Supported converters have better robustness and exhibit better performance on linear indivisible problems [16]. In 2018, KJ [17] used SVM algorithm to classify and verify the Wisconsin breast cancer (diagnosis) data set. The result showed better robustness. Hasan [18] used SVM, RFT (random Forest tree), and NBC (Naive Bayes classifier) algorithms, respectively, to establish the machine learning model based on “macromolecule postures.” The prediction accuracy of all models reached more than 82% and had good prediction performance.

There are many optimization problems in the field of medical research. Traditional optimization algorithms take the precise mathematical characteristics of the objective function as the goal [19] and have the advantages of practicality and efficiency, and their representatives include Newton's method. Traditional optimization algorithms must firstly analyze the problem itself, know the mathematical form of the optimization solution, and have certain limitations in solving problems such as multiobjective optimization and global optimal solutions. Intelligent optimization algorithm is a type of bionic algorithm that imitates nature [19], and it does not require high understanding of the optimization problem itself; it has certain advantages in global search.

The swarm intelligence algorithm is an intelligent optimization algorithm that simulates the behavior of biological swarms [20, 21]. Since Beni and Wang firstly proposed the concept of swarm intelligence in 1989, swarm intelligence algorithms have continued to develop. The mainstream algorithms include ant colony algorithm [22], particle swarm algorithm [23], fish swarm algorithm [24], firefly algorithm [25], and cuckoo Bird Algorithm [26].

The time and location of liver cancer recurrence have a serious impact on the quality of life of patients. In this paper, CS-SVM is used to predict the location of liver cancer recurrence, and SC-SVR is used to predict the recurrence time of liver cancer patients, so as to conduct timely intervention and treatment according to the recurrence situation of different patients. The traditional SVM algorithm is limited by the empirical parameters. In this paper, cuckoo algorithm is used to improve the parameters of SVM to improve the predictive performance of the traditional SVM algorithm.

The structure of this article is as follows. The first part, the introduction, introduces the process and main research content of this article. The second part, the introduction of the method, mainly introduces the basic principles of the method in this article. This article combines the optimization characteristics of the cuckoo algorithm with the SVM algorithm to implement an improved SVM prediction algorithm based on the cuckoo algorithm. The third part, an empirical analysis, mainly verifies the prediction effect of the SVM prediction algorithm based on the cuckoo algorithm on the recurrence time and location of cancer patients. At the same time, the BP neural network and logistic regression are used to predict the recurrence time and location of cancer patients and, thus, to compare the prediction effects between different algorithms.

## 2. Method Principle

Support vector machine is essentially a linear classifier with the largest interval defined in the feature space. The characteristic of the largest interval is different from other classifiers. Both this algorithm and its derivative support vector regression have good performance.

CuckooSearch (CS) is a swarm intelligence algorithm proposed by Yang et al. [26]. The algorithm is affected by the characteristics of cuckoo reproduction and combined with Levy flight to solve the optimization problem. Cuckoo algorithm is used in this paper to improve the support vector regression, which makes the prediction model parameters more suitable. In terms of breeding methods, cuckoos are different from other birds in that they do not build nests and breed offspring. Generally, they lay their eggs in the nests of other birds and their offspring are raised by the host bird. The eggs produced by cuckoos and the eggs of the host bird have little difference in appearance. If the host bird finds a cuckoo egg, it will abandon the nest and rebuild the nest. Inspired by the cuckoo's reproduction method, Yang et al. [26] proposed the cuckoo algorithm in combination with levy flight in 2009.

In the process of population update, the individual other than the optimal one in the nest will be replaced. The position of the *i*th individual in the *t*+1 iteration *s*_*i*_^*t*+1^ can be calculated by the following formula:

(1) $$\begin{array}{c} s_{i}^{t+1}=s_{i}^{t}+\alpha ⊗\text{Levy}\left(\lambda \right)⊗\left(s_{i}^{t}-s_{\text{best}}^{t}\right). \end{array}$$

Type, ⊗ said peer-to-peer multiplication, alpha > 0 as the step size parameter, and *s*_best_^*t*^ as the optimal individual, for the current population (*s*_*i*_^*t*^ − *s*_best_^*t*^) ensures the best individual will not be replaced. Levy(*λ*) is a random search path for Levy's flight, whose step length conforms to Levy's distribution:

(2) $$\begin{array}{c} \text{Levy}：\;u=t^{\left(-\lambda \right)},\;\left(1\leq \lambda \leq 3\right). \end{array}$$

The Mantegna algorithm can be used to simulate Levi's flight, and its step size formula is

(3) $$\begin{array}{c} l=\frac{u}{{\left|v\right|}^{\left(1/\beta \right)}}, \end{array}$$

where *u* and *v* follow the normal distribution: *u* ~ *N*(0, *σ*_*u*_^2^), *v* ~ *N*(0, *σ*_*v*_^2^). Among them,

(4) $$\begin{array}{c} \partial_{u}={\left\{\frac{\Gamma \left(1+\beta \right)\sin\left(\pi \beta /2\right)}{\Gamma \left[\left(1+\beta \right)/2\right]\beta \cdot 2^{\left(\left(\beta -1\right)/2\right)}}\right\}}^{\left(1/\beta \right)},\;\partial_{v}=1. \end{array}$$

Cuckoo algorithm selects the optimal solution of individual most problems through multiple iterations.

### 2.1. SVM Cancer Recurrence Prediction Algorithm Based on Cuckoo Algorithm

The nonlinear SVM and SVR models have different penalty coefficients and kernel functions, and so their prediction performance will also be different. The cuckoo algorithm has the characteristics of strong global search ability, self-organization, and parallelism [27]. Therefore, it is a feasible method to search for SVM model parameters by cuckoo algorithm to improve the performance of SVM.  Figure 1 is a flowchart of the algorithm. The steps of the SVM algorithm based on the cuckoo algorithm are given below.

1. The boundary conditions of SVM parameters are set.
2. The kernel function used in this paper is the RBF kernel function. The relevant boundary condition is *γ*, *C* ∈ [10^−3^, 10^5^], where C is the penalty term coefficient and *γ* is the parameter in the RBF kernel function.
3. Initial population.
4. Li Ming et al. conducted experiments on test function and found that the population size *N* = 15 and discovery probability *p*=0.25 can solve most problems. Therefore, this paper also uses a population size *N* = 15, a discovery probability *p*=0.25, and a search step parameter *α* = 0.1 to initialize the population.
5. The fitness value of each individual is calculated. This paper uses the mean square error MSE of SVM as the objective function value of the optimization algorithm.
6. The individual parameters with the smallest fitness value in the population are recorded.
7. It is judged whether it is less than the minimum fitness value of the previous iteration; if yes, we go to the next step; otherwise, we go to step (7).
8. The global minimum and corresponding parameters are updated.
9. It is judged whether it reaches the upper limit of iteration; if so, the optimal parameter combination is directly output; otherwise, the optimal individual is kept and the population is updated, and return we to step (3).

## 3. Empirical Analysis

### 3.1. A Sample of Cancer Patients

Hepatocellular Carcinoma (*HCC*) is one of the most common malignant tumors in the world. Clonorchiasis, alcoholic hepatitis, and viral hepatitis are the main causes [28]. The mortality rate is the second and the incidence rate of liver cancer is the fourth in China's malignant tumors according to the relevant data in 2019. [29].

Recurrence after cancer treatment is an important factor affecting the long-term survival of cancer patients. To study the influencing factors of recurrent cancer and carry out certain clinical intervention strategies can effectively improve the survival rate of cancer patients.

### 3.2. Cancer Index-Related Items and Their Weights

Six indicators including immune, tumor, microenvironment, psychological, nutritional, aerobic exercise, and advanced work were selected as predictors of postoperative recurrence of cancer patients in this paper. These indicators are determined through the investigation of doctors in relevant specialties. The number 1 is the evaluation standard of six indicators, including the related items, weight, and evaluation grade of each index.

Table 1 is the evaluation criteria of each index, including six index-related items. Weights are given according to 10 doctors' experience. According to the weights, the best score for grade A is 0.25, and the worst score for grade D is 1. The formula of comprehensive score of each index is as follows:

(5) $$\begin{array}{c} I=\frac{\sum_{i=1}^{n}x_{i}w_{i}}{\sum_{i=1}^{n}w_{i}}. \end{array}$$

In formula (5), *x*_*i*_ is the value of immune index *I* and*w*_*i*_ is the weight of the *i*-th immune indicator item. Liver cancer is a kind of common cancer. Seven hundred and seventy-six cases of liver cancer recurred after operation were collected in this paper. Among them, 520 cases recurred in situ, accounting for 67.01% of the total samples, and 256 cases recurred in other places, accounting for 32.99% of the total samples.

### 3.3. Prediction of Recurrence Time of Cancer

For the seven input indicators *X*_*i*_(*i*=1, ⋯, 7), the average score of the disease can be obtained by weighting the score of the disease.

The recurrence time of the samples collected in this paper is 1–60 months. Firstly, the recurrence time is normalized by the following formula, and it becomes a continuous variable:

(6) $$\begin{array}{c} Y=\frac{t-t_{\min}}{t_{\max}-t_{\min}}. \end{array}$$

The 776 collected training sets and test sets are randomly generated according to the ratio of 7 : 3. The specific implementation method is to randomly generate 776 random numbers evenly distributed between 0-1. If the *i*-th number is greater than 0.3, the *i*-th sample will be classified as the training set; otherwise, it will be classified as the test set.

This paper uses libsvm software package based on the University of Hong Kong. The cuckoo algorithm takes the mean square error of the test set as the fitness function. The mean square error is calculated as follows:

(7) $$\begin{array}{c} \text{MSE}=\frac{1}{n}{\sum_{i=1}^{n}\left(y_{i}-{\hat{y}}_{i}\right)}^{2}. \end{array}$$

The initial parameters of cuckoo are shown in Table 2.

Firstly, the SVR cancer recurrence time prediction model based on cuckoo algorithm optimization was established by normalizing the recurrence time, and the best penalty coefficient is *C*=2.9697*∗*10^14^. The kernel function parameter is *g*=37.6832 and the final mean square error is 9.2101.  Figure 2 shows the recurrence time prediction chart of the SVM test set.

BP neural network is a concept proposed by Rumelhart and McClelland in 1986. It is a relatively basic neural network. The BP neural network has excellent nonlinear fitting performance. Therefore, this section intends to use BP neural network algorithm to predict the recurrence of liver cancer patients after operation and compare the two fitting effects.

The BP neural network used in this paper is based on MATLAB software built-in neural network toolbox function, Table 3 shows the basic parameters of BP neural network, and Figure 3 shows the change image of mean square error (MSE) of the BP neural network iteration process.

From Figure 3, we can see that the BP neural network has been iterated for 800 times. At 200 times, the MSE of test set, training set, and verification set have become stable, and the MSE is 177.9451.

Figure 4 shows the prediction chart of recurrence time of the BP neural network, and the mean square error is 177.9451. Compared with Figure 2, the prediction effect of cancer recurrence is poor.

### 3.4. Prediction Model of Recurrence Location of Hepatocellular Carcinoma Based on SVM

The location of cancer recurrence can be divided into in situ recurrence and other site recurrence. The 776 collected training sets and test sets were randomly generated according to the ratio of 7 : 3. The specific implementation method is to randomly generate 776 random numbers evenly distributed between 0 and 1. If the *i*-th number is greater than 0.3, the *i*-th sample will be classified as the training set; otherwise, it will be classified as the test set.

In cuckoo search algorithm, the prediction accuracy of test set samples is taken as the fitness function. The initial parameters of cuckoo are shown in Table 4:

This experiment establishes a prediction model for the recurrence location of SVM cancer based on the cuckoo algorithm optimization. After 250 iterations, the optimal penalty factor is *C*=7.29*∗*10^14^, kernel function parameter *g*=7.07*∗*10^3^, and the prediction accuracy of test set samples was 94.39%.  Figure 5 shows the predicted test set classification and the actual test set classification. It can be seen from the figure that in situ recurrence is almost completely predictable; however, the accuracy of it at this site is low.

Table 5 shows that, for in situ recurrence, the model has a good prediction accuracy of 97.5%, 84.4% for other site recurrence, and 93.1% for the whole population.

Figure 6 shows the ROC curve of cancer recurrence location based on SVM. Table 5 shows that the overall sample prediction accuracy is 95.7%. The ROC curve shown in Figure 6 is more to the upper left with AUC 0.95, and the model performs well.

Normally, the main multivariate statistical methods to deal with qualitative variables are logistic regression analysis, discriminate analysis, and probit analysis. Among them, logistic regression analysis is widely used in practice. This section uses a binary regression model to fit and predict the recurrence location of cancer.

Table 6 fits parameter results based on a full sample data model of seven factors, indicating that baseline finger symptoms, nutritional finger symptoms, aerobic exercise, and advanced work are positively correlated with relapse at the other recurrence, while the remaining factors are negatively correlated with relapse at the other recurrence.  Table 7 is the overall sample prediction table.

As shown in Table 7, the overall accuracy of logistic regression is low, only 63.14%, which is much lower than that of SVM.

Figure 7 shows a logistic-based ROC curve for the location of cancer recurrence.  Table 7 shows that the overall sample prediction accuracy is 63.14%. The ROC curve in Figure 6 is more to the upper left, and the AUC is 0.64. The performance of the model is general.

## 4. Conclusions

The length of postoperative recurrence time plays an important role in the quality of life and living standard of patients with liver cancer. The study of recurrence time and recurrence location of patients with liver cancer has a crucial impact on postoperative intervention. This paper proposes an SVM recurrence prediction model based on cuckoo optimization algorithm.

Firstly, the general problems and solutions of support vector machine are introduced. At the same time, a kernel function is introduced to solve the problem of nonlinear fitting. Secondly, the basic idea of cuckoo algorithm is introduced, and an improved support vector machine model is proposed by combining cuckoo algorithm with support vector machines (SVMs).

Then, the status of patients with recurrence was evaluated, and the factors influencing the recurrence of cancer patients were divided into seven modules: basic indications, immune indicators, tumor indications, nutritional indicators, psychological indicators, microenvironment indicators, aerobic exercise, and advanced work. The score of each module is the weighted average of the scores of related items of each module.

Finally, the experimental verification is given. According to 776 cases of liver cancer recurrence samples collected, the recurrence time and recurrence location are predicted, respectively. The mean square error of recurrence time prediction was 9.2101, which was far less than 177.9451 of the BP neural network; the accuracy of recurrence location prediction was 95.7%, which was much higher than 63.14% of logistic regression. Experiments show that the improved SVM model based on cuckoo can effectively predict the recurrence time and location of cancer. Meanwhile, our finding indicated that this predication method can also be applied to other kinds of cancer in terms of rate or site of recurrences.

In the future work, we will study the mechanism of liver cancer recurrence, other cancer recurrence, and the related signs in this paper and also pay attention to the application of new machine learning algorithm.

## Figures and Tables

**Figure 1:** SVM algorithm parameter optimization flowchart.

**Figure 2:** Prediction of recurrence time of SVM.

**Figure 3:** MSE iterative graph of the BP neural network.

**Figure 4:** BP neural network recurrence time prediction chart.

**Figure 5:** SVM test set classification prediction diagram.

**Figure 6:** ROC curve of cancer recurrence location based on SVM.

**Figure 7:** Logistic-based ROC curve for cancer recurrence location.

**Table 1:** Correlation terms and weight of cancer indications.

Indications	Associated items and their weights
Basic indications	Systemic diseases, 2; family history of cancer, 2; necessary dependence, 3; age, 1; obesity, 1; habitual high risk, 1; regional high risk, 1

Immune indications	CD3+CD4+CD8+/CD45+, 4; CD3+CD4+/CD45+, 8; CD4+/CD8+, 10; CD3+CD16+CD56+/CD45+, 6; CD3-CD56+,5; CD4+CD25+, 1; exercise electrocardiograph (X ± SD), 2; exercise electrocardiography (X ± SD), 2

Tumor indication	Size, 10; space occupying, 10; invasion, 10; angiogenesis, 10; pathological classification, 3; CTC value, 9; differentiation, 10; mutation target, 1

Nutrition indication	Total nutrition, 6; balanced nutrition, 3; nutritional safety assessment, 5; cancer cell proliferation, 10; immune cell proliferation, 10; angiogenesis, 8; amino acid assessment, 5; proteomic assessment, 10

Mental indication	Life event scale, 1; cornell medical index, 2; self-rating anxiety scale, 5; self-rating depression scale, 5; Beck Anxiety Scale, 5; Beck Depression Questionnaire, 5; Pittsburgh sleep quality index, 4; Texas social behavior questionnaire, 3; family function assessment, 1; exercise electrocardiograph (X ± SD), 2

Microenvironment indication	O2, 3; PH value, 4; interstitial pressure, 2; inflammatory response, 7; vascular permeability, 6; CTC value, 9; protein mass spectrometry, 8

Aerobic exercise and advanced work	Aerobic exercise, 4; advanced social work, 3; Texas social behavior questionnaire, 3

**Table 2:** Experimental conditions.

Parameter name	Parameter value
Number of iterations, T	250
Population size, N	15
Probability of discovery, P	0.25
Step, *α*	0.1
Penalty parameter C bounds	[0.01, 10^15^]
Kernel function parameters, g	[10^−14^, 10^5^]

**Table 3:** BP experimental conditions.

Parameter name	Parameter value
Maximum number of iterations	1000
Minimum error	0.00001
Learning rate	0.000001
The first hidden layer	10
The second hidden layer	20

**Table 4:** Experimental conditions of SVM.

Parameter name	Parameter value
Iterations number, *T*	250
Population number, *N*	15
Probability of discovery, *P*	0.25
Step length, *α*	1
Penalty parameter C bounds	[0.01, 10^15^]
Kernel function parameter, g	[10^−14^, 10^5^]

**Table 5:** Full sample prediction situation.

Measured value predicted value	Original site	Other site	Percentage
Original site	507	13	97.5
Other site	20	236	92.1
Percentage			95.7

**Table 6:** Logistic regression coefficient table.

	*β*	Standard error	Wald	Significance
Basics	0.49	0.040	144.4	<0.001
Immunity	−0.16	0.013	157.5	<0.001
Tumor	−0.07	0.008	76.7	<0.001
Nutrition	0.04	0.009	15.4	<0.001
Psychology	−0.11	0.013	66.8	<0.001
Microenvironment	−2.13	0.424	25.2	<0.001
Advanced quantity	0.12	0.029	17.1	<0.001
Constant quantity	−2.74	.595	21.2	<0.001

**Table 7:** Overall sample prediction table.

Measured value predicted value	Original site	Other site	Percentage
Original site	468	52	90.0
Other site	234	22	8.59
Percentage			63.14

## Data Availability

The data used to support the findings of this study are available from the corresponding author upon request.
